# An Improved Convolutional Neural Network-Based Scene Image Recognition Method

**DOI:** 10.1155/2022/3464984

**Published:** 2022-06-29

**Authors:** Pinhe Wang, Jianzhong Qiao, Nannan Liu

**Affiliations:** ^1^School of Computer Science and Engineering, Northeastern University, Shenyang 110169, China; ^2^China Coal Technology Intelligent Storage and Loading Technology Co, Ltd., Beijing 100013, China

## Abstract

To solve the problems existing in the research of scene recognition, this paper studies a new convolutional neural network target detection model to achieve a better balance between the accuracy and speed of high-speed scene image recognition. First, aiming at the problem that the image is easy to be disturbed by impurities and poor quality in fine-grained image recognition, a preprocessing method based on the Canny edge detection is designed and the Canny operator is introduced to process the gray image. Second, the L2 regularization algorithm is used to optimize the basic network framework of the convolutional neural network, enhance the stability of the model in a complex environment, improve the generalization ability of the model, and improve the recognition accuracy of the algorithm to a certain extent. Finally, by collecting the campus environment datasets under different environmental conditions, the location recognition experiment and heat map visualization experiment are carried out. Experiments show that compared with the basic convolution neural network algorithm, the algorithm has better recognition performance and good generalization ability. The research of this study realizes the effective combination of multiframe convolution neural network and batch normalization algorithm and has a good practical effect on scene image recognition.

## 1. Introduction

Artificial intelligence is an important branch of computer science, and the study of artificial intelligence aims to make machines think and humanly react to the outside world so that they can perform complex tasks that are beyond the reach of humans [1]. In recent years, as scientists have continued to study the field of computational science, more specialized computer system programs have emerged, and the scope of AI applications has continued to expand. Nowadays, artificial intelligence is developing toward comprehensive applications in multiple fields, and it not only has significant advantages in various deterministic information processing fields but also has gained wide attention in important fields such as computer vision and machine translation [2]. The means and methods used by human beings to receive and acquire various external information in life mainly include vision, hearing, taste, touch, etc., and more than 80% of the information is considered to be received and acquired through various human visual methods. Therefore, vision is widely considered to be the most important means of acquiring and receiving information in the world nowadays. Nowadays, computer vision systems, as an important part of modern artificial intelligence, aim at understanding and analyzing the image content automatically by using computers and computers to perform various computer vision tasks such as object detection, recognition, and tracking. The saliency detection algorithm used in this study can well eliminate the background interference of the image and input more semantic information about the salient target contour into the neural network.

As an important research direction in the field of image processing, image recognition is the most basic task of computer vision and the basis of various other vision tasks. The research of image recognition technology started in the 1940s, and with the emergence of artificial intelligence technology, image recognition technology has been rapidly developed. For example, in the field of autonomous driving, the use of cameras to distinguish obstacles such as trees, animals, and pedestrians in front of the driver can effectively help drivers avoid hazards [3]. The image dataset is an important driving force in the development of image recognition, which contains 15 million images and more than 20,000 categories. The ImageNet dataset contains data from 15 million images and more than 20,000 categories. The emergence of the ImageNet Large-Scale Visual Recognition Challenge (ILSVRC) based on this dataset has facilitated the rapid development of deep learning algorithms in the field of image recognition, achieving results that far exceed those of general image recognition algorithms based on manual feature extraction, and the emergence of several algorithms such as AlexNet, ResNet, InceptionNet, and other classic deep learning-based recognition algorithms. At the last edition of the competition in 2017, ImageNet announced the end of a large vision challenge based on this dataset and will henceforth work on solving unsolved vision challenges. In this competition, SENet took the top spot in this image recognition with a top-5 error rate of 2.25%, which has far surpassed human ability and shows the maturity of image recognition technology [4].

However, if the units of the values on the vector dimension differ by a large order of magnitude, standardization is required; otherwise, the difference calculation of a certain dimension will be missing in the result. The advent of artificial neural networks has given rise to an unprecedented ray of hope for learning deep learning. Artificial neural networks are not a recent term; they have been around since the 1850s. The reason it has not been generally accepted by humans until recent years is that computers can store more data and many datasets have been specifically developed for the study of neural networks. As these datasets became higher and higher quality, there was a desire to have an algorithm that could discover the nature of things from massive amounts of data [5]. The second is the emergence of large-scale models. After decades of development, models are now becoming increasingly like the human brain, with many connected neurons inside them. Scientists expect this growth to steadily continue in the coming years. Finally, the training power of AI convolutional neural network models continues to improve, and the accuracy of recognition on each large data set continues to improve. Deep learning is rapidly evolving, but it is still in its infancy, and its applications in many areas have not yet been fully developed by humans.

In view of this, this study studies a new convolutional neural network target detection model to achieve a better balance between the accuracy and speed of high-speed scene image recognition. The specific work is as follows:

1. Aiming at the problem that the image is easily disturbed by impurities and poor quality in fine-grained image recognition, a preprocessing method based on the Canny edge detection is designed, and the Canny operator is introduced to process the gray image
2. The L2 regularization algorithm is used to optimize the basic network framework of the convolutional neural network, which enhances the stability of the model in a complex environment, improves the generalization ability of the model, and improves the recognition accuracy of the algorithm to a certain extent
3. By collecting campus environmental datasets under different environmental conditions, the experiments of location recognition and heat map visualization are carried out

The remainder of this study is organized as follows. In the next section, the related works will be shown in detail. In Section 3, the scene image recognition method based on an improved convolutional neural network is studied. In Section 4, the simulation and experiments are carried out. Finally, some conclusions are drawn in Section 5.

## 2. Related Works

Researchers in the field of computer vision have been focusing on the recognition of images. Image recognition is a subjective process, and even an untrained child can easily identify a target by looking at the different colors, sizes, and dimensions in a picture. But when the computer receives these RGB pixel matrices, it cannot directly capture the shallow features of the image, let alone localize them. Also, factors such as different image shapes and blurred distinctions between images and backgrounds can make the recognition of images very difficult [6]. Traditional image recognition operates feature extraction and image classification separately, which makes it necessary to construct features for image extraction by a human. This not only increases the human workload but also greatly reduces the efficiency of image feature extraction. When faced with feature extraction of some complex images, people tend to ignore most of the details, such as color, texture, lightness of the image, and some other shallow features [7]. This will greatly limit the application scenarios of traditional image recognition. In recent years, the application of convolutional neural networks started to be popular, and from the appearance of the AlexNet convolutional neural network in 2012 to the Mask R-CNN algorithm proposed by Cong I, the convolutional neural network started to become practical. Its most important feature is that feature extraction and classification are integrated into a single neural network [8]. Convolutional neural networks integrate the feature extraction function into a multilayer perceptron by reorganizing the structure, reducing its weight, and eliminating the complex image feature extraction process before recognition. The tight connections between layers within the network allow the convolutional neural network to process images better, while at the same time it can actively extract some useful and relevant features from the data. This phenomenon is called gradient explosion. The reason for the exploding gradients is a covariant shift within the network. With the batch normalization (BN) algorithm, we can maximize the guarantee that each forward pass output is on the same distribution.

The convolutional neural network (CNN) is inspired by the study of the cat visual cortex and can be considered a masterpiece of bionics. A convolutional neural network is a kind of neural network originally designed for image recognition, and its main feature is the sharing of local receptive fields and weights. These features not only reduce the computational effort of the neural network but also improve its robustness [9]. This network structure makes great use of the spatially interconnected nature of images and is highly invariant to translation, scaling, skewing, or co-otherwise forms of distortion. Most importantly, the convolutional layers can be viewed as an adaptive feature extraction scheme [10]. The accumulation of many convolutional layers allows convolutional neural networks to progressively upgrade features from a low level, and even pixel level, to a high level. Zhou proposed to use a pretrained convolutional neural network for location recognition and experimentally demonstrated that compared with traditional manual features, the features extracted by the convolutional neural network can achieve better recognition performance when the environmental appearance conditions change [11]. Dhillon and Verma used the AlexNet network proposed by Krizhevsky l20 to experimentally analyze the performance of different layers of the convolutional neural network when the environmental conditions change and the viewing conditions change [12]. Yadav and Jadav added a new pooling layer at the output of one of the layers of the convolutional neural network, which was implemented by employing a local aggregation feature description, the parameters of this pooling layer could be trained in an end-to-end manner, and this pooling layer was also called the NetVLAD layer [13].

Scholars at home and abroad have conducted a series of research studies on the intersection of convolutional neural networks and image recognition, and have made great progress in face recognition, character recognition, remote sensing image recognition, and traffic sign recognition. However, the current research on the application of convolutional neural networks to complete the image recognition of urban scenes is not perfect, and it cannot adapt well to the complex environment, such as the situation where the light changes drastically and the obstacles obscure the feature points, while there are still some problems in the recognition accuracy, and there is room for improvement [14]. Therefore, this study makes a series of improvements to the convolutional neural network to adapt it to the complex environmental changes in urban scenes and accomplish the image recognition with high accuracy and good real time, which has certain research significance.

## 3. Research on Improved Convolutional Neural Network-Based Scene Image Recognition Algorithm

### 3.1. Improved Convolutional Neural Network-Based Algorithm Design

In the era of continuous development of deep learning, the model of combining deep learning and attention mechanism becomes more important, because the neural network based on attention mechanism not only shows its strong autonomy in the learning of attention but also humans can improve the understanding of neural network with the help of attention mechanism. When the convolution kernels of head, body, and tail are set with 2048, 4096, and 2048, respectively, the TPA-CNN algorithm achieves the best recognition effect. The attention mechanism requires the help of a mask (mask), which is carried out in the image with another layer of weights to identify the key features of the original image and then learn these key features that are attended to in the network, that is, the formation of attention [15]. This model produces two types of attention: soft attention (soft attention) and strong attention (hard attention). The former attention is deterministic, focusing on the region and channel features of the information, and its process is simple, usually, after the training is completed and then passing through the grid. The most important feature of soft attention is its differential nature, and the computation of gradients can be performed by forward and backward propagations.

The spatial transformer network (STN) model was published in NIPS in 2015 as a representative of the soft attention mechanism, and its principle is to replace the spatial information between the input image and another space, and then compress the feature information in the network by applying maximum pooling or mean pooling in the pooling layer of the convolutional network, thus achieving the effect of reducing the computation and thus improving the recognition accuracy. This not only preserves the key information but also reduces the amount of computation and improves the recognition accuracy. The spatial transformer module in the STN network model can identify the region of the image to be focused on, while the spatial transformer module can rotate, scale, and zoom the image. The transformer module has the functions of rotation, scaling, and transformation so that the important local information of the image can be extracted by transformation. As shown in Figure 1, the STN network uses maximum or average pooling in its pooling layer to compress the feature information in the convolutional neural network, thus reducing the number of operations in the neural network and improving the image recognition accuracy.

In general, the data input to the convolutional neural network is a color image with three channels of RGB, so we generally process the original data by convolving it with three convolutional kernel filters that can be trained to obtain the mapping layer on *C*1. Then, the ReLU activation function is used to process the convolved image features to further highlight the complex feature information of the image to obtain the mapping layer on *S*2. The pooling operation of the pooling kernel then selects and filters the processed features to obtain the feature information mapping map on *C*3. The information map on *C*3 is then processed and transmitted to the *S*4 layer, and the pixels in the *S*4 layer are transmitted to other neural networks later by the nonspatial expansion structure of the fully connected layer to generate one-dimensional signals.

(1) $$\begin{array}{c} U_{i}^{j}=\sum_{i\in M_{j}}^{N}x_{l}\times W_{ij}^{l-1}+2b,\\ x_{l}=f\left(x\right)+f\left(U_{i}^{j}\right). \end{array}$$

The structure of a convolutional neural network contains several implicit layers, and these implicit layers include millions of parameters, and the training of these parameters needs to learn through a large amount of image data, and implicitly learn experience and knowledge from these large amounts of image data, so that the features extracted by the convolutional neural network can effectively extract multiple layers of visual information with different contents from the original image, and after multiple layers of nonlinear transformation [16]. The multilayer nonlinear transformation and the extracted features also have powerful nonlinear transformation ability, which can effectively distinguish various changes in the environment, such as lighting, weather, and seasons, to obtain more advanced information and ensure that the extracted features have outstanding invariant advantages in complex environments. The feature extraction algorithm is used to obtain the feature vector of the image after feature extraction, and then, the distance between the query image and the feature vector of the reference image is calculated to determine whether a match occurs, and the closer the distance is, the more the two images match, and then, a threshold is set to calculate the accuracy rate of the whole location recognition algorithm and other parameters. At present, the more commonly used methods to calculate the sample distance in the research of image recognition and image classification are Euclidean distance, cosine distance, Manhattan distance, etc.

(2) $$\begin{array}{c} \text{Manhanttan\_dist}=\sum_{i=1}{\left|y_{i}^{2}-x_{i}^{2}\right|}^{\sqrt{2}},\\ f_{\max}\left(v\right)=y^{2}-\underset{1<M\leq \text{t}}{\max}v_{M}. \end{array}$$

Euclidean distance can be used to calculate two vectors with complete data and no missing dimensional data, i.e., if the units of measurement between the two vector dimensions are the same, there is no problem to use this formula, but if the units of the values in the vector dimensions differ by a large order of magnitude, it is necessary to do the normalization process; otherwise, it will result in the calculation of the difference of a missing dimension. All dimensions of the vector are separately treated so that each dimension satisfies the standard normal distribution. The flow of the improved deep convolutional neural network algorithm is shown in Figure 2.

### 3.2. Scene Image Recognition Algorithm Model Construction

The scene recognition method designed in this chapter first needs to do a preprocessing operation on the scene images in the training dataset to get a consistent size image set, then the processed images are passed through a convolutional neural network to get the global features of the image, then, on the one hand, the global features are the global representation of the whole scene image, which are input to a fully connected layer, and on the other hand, several features are adaptively selected from the global feature map, which is treated as vertices of the graph structure in the form of feature vectors and input to the graph neural network. Finally, the two results are connected and fed into a fully connected layer and a softmax layer for scene classification, and the model is iteratively trained until the whole model converges and is saved. After the training is completed, the scene classification system is tested and the input image is the result of the category obtained by the classification. The graph neural network is a ConvGNN network, and the graph pooling module is a GSAPool-based pooling method.

(3) $$\begin{array}{c} x_{i}^{*}=m_{i}s_{i}+\frac{x_{i}+m_{i}}{s_{i}-m_{i}}. \end{array}$$

The superpixel images segmented by the SLIC algorithm are used as the basis to build absorbing Markov chains to establish connections between all superpixel clustering centers. Markov chains are discrete-event stochastic processes with Markovian properties, where at each node, the system can convert from one state to another or maintain the current state according to probability [17]. To achieve the purpose of eliminating drift errors, image recognition of marker position nodes using the convolutional neural networks will inevitably require the high accuracy of CNN models. In practical applications, the target scenes are often more or less different from the image set at the time of training, and how to make the model maintain good adaptability and accuracy in complex environments is the issue focused on in this study. The specific workflow of dropout is as follows: without changing the input and output of the original model, some neurons are randomly selected to “die,” and the rest continue to work, thereby greatly reducing the parameters involved in the calculation.

(4) $$\begin{array}{c} \text{dist}=\sum_{i=1}^{N}\left(\frac{s_{i}}{x^{2}+y^{2}}\right). \end{array}$$

To address the problem that the number of collected scene images is not enough to support the neural network training, this study adopts a data enhancement algorithm to increase the diversity of the training set from two perspectives of geometric transformation and color space transformation, so that the neural network can learn more features in different scenes and improve the recognition accuracy of the model. To highlight the salient target effective information of the image in the training phase of the CNN model, while suppressing the interference information, the saliency detection algorithm used in this study can well eliminate the image background interference and input more semantic information about the salient target contour into the neural network. The improved convolutional neural network-based scene image recognition algorithm is proposed in this study, and the specific structure is shown in Figure 3.

The performance of a deeper network is not necessarily better. Using a deep convolutional network with a common architecture, the error rate of a 56-layer network is higher than that of a 20-layer network. The effect of a different number of convolutional kernels on the performance of the TPA-CNN algorithm in the channel fusion operation is experimentally verified.  Figure 4 shows the effect of choosing a different number of convolutional kernels on the recognition accuracy. The horizontal coordinates indicate the total number of convolutional kernels, and the height ratios of different colors in the bars corresponding to each coordinate indicate the percentage of the number of convolutional kernels in the head, body, and tail in the MCAF module. The vertical coordinates in the figure indicate the recognition accuracy of different convolutional kernels on the CUB-200-2011 bird dataset. As shown in Figure 4, when the number of convolution cores of the MCAF module is half or twice the number of 1M, 2M, and 3M channels of the input characteristic diagram, the recognition accuracy of the CUB-200-2011 dataset will be reduced. In TPA-CNN algorithm, when the convolution kernels of head, body, and tail are set to 2048, 4096, and 2048, respectively, the best recognition results are obtained.

If too many parameters are generated in the process of training the model and too few training samples, the phenomenon of overfitting can easily occur. The main manifestation is that the network can show high recognition accuracy on the training image set with little difference from the real value, while the recognition accuracy on the test image set decreases. To solve this problem, the dropout strategy is introduced after the fully connected layer [18]. The dropout works by randomly selecting some neurons to “die” without changing the input and output of the original model, and the rest to the fully connected layer of the VGG network uses a 1 × 1 convolutional kernel several times. First, its dimensionality can be consistent with the original fully connected structure. Second, the 1 × 1 convolutional kernel does not focus on the local information of the feature map when performing feature extraction but focuses on the information integration of the feature map. In addition, when the number of convolutional kernels reaches a certain level, it is very time-consuming to perform convolutional operations, and then, the computational complexity can be reduced by using small convolutional kernels. It can correct a target object to make it easier to recognize by rotating, panning, zooming in, and zooming out, or even extracting it separately to fill a screen, and then inputting it into the neural network for recognition.

The algorithms in this study can achieve an accuracy of more than 90% on different datasets and can adapt to the changes in image angle, occlusion, and illumination in complex environments. The SeqSLAM algorithm is more robust in recognizing the images in the Nordland dataset with obvious seasonal changes, but the proposed algorithm achieves good results. For the NUC dataset and Garden Point dataset, the algorithm in this study shows great advantages, and the accuracy rate is higher than the other three algorithms, as shown in Figure 5.

Strongly supervised recognition algorithms require a large amount of manual annotation information and consume more human and material resources. To solve the above problems and meet the practical needs, in this chapter, we propose two weakly supervised information-based image recognition methods for fine-grained image classification [19]. One is a joint residual network and inception network to improve the ability to capture fine-grained features by optimizing the network structure of convolutional neural networks. The other is an improvement of the bilinear CNN model with feature extractors selected from the Inception-v3 module and Inception-v4 module proposed by Google, and finally, different local features are pooled together for classification. One of the major principles of deep learning is that the deeper the neural network is, the better the expressiveness of the network. But extremely deep networks are not easy to train, and the network performance may also degrade when the network reaches a certain depth. From 2012 to 2014, the number of layers of neural networks grew from 8-layer AlexNet to 19-layer VGG, hitting a bottleneck where gradient disappearance and gradient explosion had been a problem for researchers. In 2015, Versaci and Morabito proposed a deep residual network that allows the error rate of the network to decrease with depth and won the ImageNet 2015 competition by a wide margin [20]. Therefore, the learning integrates the features extracted from the three convolutional layers Conv3, Ccmv4, and Cmw5, which contain relatively rich semantic information and high-level information in HybridNet, and from the experiments in Chapter 3, the three convolutional layer features are in the position. It shows better robustness in recognition.

## 4. Analysis of Results

### 4.1. Feasibility Analysis of the Improved Convolutional Neural Network-Based Algorithm

The entire target localization module is performed on the global feature map extracted from the feature extraction module *F*_*x*_, which contains deep semantic information, has fewer parameters compared with the original map, and has higher training efficiency. Spatial transformer networks (STNs) are used in the target localization module. In the training of neural network models, the same target may have different angles and sizes, which may affect the classification results. Therefore, the STN network was born, which can correct a target object to be more easily recognized by rotating the target area in the image by panning, zooming in and out, or even extracting it separately to fill a screen alone and other operations, and then input it into the neural network for recognition. The STN network can be inserted behind any layer of the convolutional neural network, not only for the input image but also for the feature map. Vision is widely considered to be the most important means of acquiring and receiving information in the world.

Before formally using convolutional neural networks for image feature learning, some important parameters need to be set. If the learning rate is too large, it may lead to model oscillation, and if it is too small, it will lead to slow parameter update and thus slow model convergence [21]. The weight decay coefficient represents the parameter in the *L*2 regularization method, and the momentum represents the parameter change per update. In this study, the learning rate is assigned to 0.001, the weight decay coefficient is assigned to 0.005, and the momentum is assigned to 0.9. If only the attention of a specific layer of features is learned, the learned attention cannot fully represent the information in the image, i.e., the imaginary information in the image is easily lost, so the attention of Conv3, which is a fusion of HybridNet with rich semantic and high-level information, is learned. Therefore, the features extracted from Conv3, Ccmv4, and Cmw5 convolutional layers, which contain richer semantic and high-level information in HybridNet, are learned, and it can be seen from the experiments in Section 3 that these three convolutional layer features show better robustness in location recognition. The algorithm proposed in this study (three-layer attention) is compared with AlexNet and HybridNet algorithms. In addition, this study also compares one-layer attention, which only uses a contextual attention mechanism in the Conv5 layer. First, the accuracy-recall curves are used to evaluate the recognition results on three publicly available datasets.

As shown in Figure 6, the accuracy-recall performance of AlexNet, HybridNet, and the proposed algorithm (three-layer attention) are comparable and the AUC is not much different in the St Lucia dataset where there are variations in lighting conditions; on the Synthesized Nordland dataset, where there are variations in seasonal conditions, the accuracy-recall performance of AlexNet and the proposed algorithm (three-layer attention) is still significantly lower and the AUC is almost constant. The accuracy-recall performance of AlexNet significantly decreases, while HybridNet and the proposed algorithm (three-layer attention) still have better accuracy-recall performance. In the Gardens Point dataset, when the lighting conditions and viewing angle conditions change, the accuracy-recall performance of AlexNet and HybridNet networks decreases significantly, while the accuracy-recall performance of the proposed algorithm (three-layer attention) is stable. This indicates that the interference of changing appearance conditions and changing viewpoint conditions in the environment can be better overcome by using the attention mechanism. It can also be seen that the recognition effect of using one layer of attention is not as good as that of three-layer attention. This makes the feature extraction of images need to be manually constructed. This not only increases the workload of human beings but also greatly reduces the efficiency of image feature extraction.

The goal of the GNN graph neural network is to update the feature values of all edge nodes by learning information about each node and edge in a network. We denote graph data by *G*(*V*, *E*), where *V* denotes the set of vertices in the graph data, *E* denotes the set of edges in the graph data, and we denote the relationship between vertices and edges by an adjacency matrix. The GNN network used in this study is the graph convolutional neural network (GCN), which maps the convolutional neural network idea used in images to the graph structure, and it can train the node features and edge-node relationship information in the graph structure end-to-end, and hierarchically extract the features in the graph structure, and each is extracted. The essence of GCN is to update the features of the graph structure, which is also a process for extracting features, and there are two main approaches to GCN: the first is the spatial approach (GCN), which aggregates and inherits RecGNNs by graph structure information.

The convolutional neural network was originally a kind of neural network specially designed for image recognition, and its main feature lies in the sharing of local receptive fields and weights. These features not only reduce the computational complexity of the neural network but also improve its robustness. For the three structures proposed, the parameters are initialized using a hybrid Gaussian model. Since they are based on Inception-v3, the same convolutional layers in the network are initialized using the pretrained Inception-v3 network from the ILSVR2014 classification dataset. Using the PyTorch deep learning framework as the training platform, the network was trained on Google Colab, a GPU server provided by Google, and trained using the RMSProp optimizer with a decay factor of 0.9. The RMSProp adds a decay rate to AdaGrad, and unlike the AdaGrad algorithm, it does not sum the previous, and it does not sum all the gradient squares, but it adds a decay rate to make it smaller. It uses a sliding average method, where the more advanced the gradient is, the less it affects the adaptive learning rate, thus avoiding the problem of decreasing the learning rate of AdaGrad more effectively and helping the network model to converge faster.

Initially, the learning rate was scaled down to 0.94 times, the original rate after 2 epochs of training using hyperparameters. The loss curve on the Stanford Cars dataset is shown in Figure 7.

### 4.2. Scene Image Recognition Algorithm Testing

In this section, we use the cross-entropy loss function for multiclassification to control the optimization of the scene image classification task. The cross-entropy loss function describes the distance between two probability distributions, and the smaller the cross-entropy is, the closer the two are to each other. The accuracy of our method is 5.4% higher than PlusNet 205 network, 5.2% higher than PlusNet 365 network, and 5.9% higher than HybridNet 1365 network. Among them, to verify that the strategy of using iterations to discover target localization regions in this study is all effective, we compare the classification probability in each iteration cycle, and the comparison results are shown in Figure 8. With the increase in the number of iterations, the model has an initial classification probability of 83.76% in the SUN 20 dataset, and the accuracy improves by 3.13% after one iteration and increases to 89.96% after three iterations, which achieved a relatively good result. The information graph on C3 is processed and transmitted to the S4 layer, and the pixels in the S4 layer are passed through the nonspatial expansion structure of the fully connected layer to generate a one-dimensional signal for transmission to other neural networks behind.

Using the test set images of each class of scene images for input, the actual output is compared with the test set sample labels to judge whether the recognition results are correct or not, all the scene recognition results are counted, and the average accuracy rate finally obtained is 62.3%. Since a total of 67 categories of scene images were recognized, 10 categories of scene images were randomly selected for this experiment, and the ratio of the training set to test set was 9 : 1. The vertical axis is the actual category of input images, and the horizontal axis is the scene recognition results of the experimental output. The average accuracy rate is 66.0%. The main reason for the error is that certain categories of scenes contain similar objects, which may confuse, for example, the bathroom and prison cell both have sinks and other sanitary ware, the buffet and meeting room both contain tables and chairs, the museum contains complicated items that may lead to confusion, etc., resulting in certain correlation and similarity. In addition, some of the scene images are blocked and stretched, which hinders the accuracy of object detection and thus affects the final scene detection results.

The improved bilinear CNN is even better than the previous strongly supervised recognition algorithm and may achieve better results if a feature extractor with better feature extraction capability is chosen. For the proposed single network model ResNet-Inception, the different stacking numbers and stacking order of modules A, B, and C have a great impact on its performance. As shown in Figure 9, the recognition performance of the three modules with different stacking orders on the CUB-200-2011 bird dataset is shown. The network achieves the best performance when the stacking order is A-B-C, and verifies that modules B and C are not suitable to be placed at the front of the network.

The above experimental results show that the proposed two weakly supervised recognition algorithms achieve better performance on both datasets. Among them, the performance of the ResNet-Inception model not only has the advantages of the inception network and residual network, but also has better recognition accuracy than the single residual network and inception network, and the recognition effect is comparable to the strongly supervised fine-grained recognition algorithm.

## 5. Conclusions

This study presents an improved urban scene recognition method based on the convolutional neural network. In this study, a TensorFlow-based framework is built from the structure-optimized VGGNet model, and the algorithm is ported based on the Xavier module, with an accuracy of 84.5% on the NUC dataset. The L2 regularization method is used to improve the structure of the neural network, enhance the portability of the algorithm, and prevent overfitting. Aiming at the problem of low accuracy of scene recognition, an image detection algorithm based on saliency is designed to eliminate the background information in the image, highlight the effective features of the image, and reduce the interference caused by illumination change and perspective change in the process of recognition. Through experimental verification and analysis, the recognition accuracy of the algorithm on the NUC dataset is improved from 84.5% to 95.3%. At the same time, we use the cross-entropy loss function for multiclassification to control the optimization of the scene image classification task. The accuracy of this method is 5.4% higher than PlusNet 205 network, 5.2% higher than PlusNet 365 network, and 5.9% higher than HybridNet 1365 network. In the future research, we can further improve the recognition accuracy and obtain higher-quality recognition results on the basis of improving the speed of the algorithm.

## Figures and Tables

**Figure 1:** Simple structure of the STN network model.

**Figure 2:** Improved convolutional neural network algorithm model.

**Figure 3:** Improved convolutional neural network-based scene image recognition algorithm.

**Figure 4:** Effect of the number of filter cores of the improved convolutional neural network module.

**Figure 5:** Image recognition accuracy of each algorithm.

**Figure 6:** Accuracy-recall relationship curves.

**Figure 7:** Loss curve.

**Figure 8:** Classification accuracy of scene image recognition model for three iteration cycles.

**Figure 9:** Recognition rate results under different combinations.

## Data Availability

The data used to support the findings of this study are available from the corresponding author upon request.
